# Potential Role of Natural Products to Combat Radiotherapy and Their Future Perspectives

This article has been retracted.

**DOI:** 10.3390/molecules26195997

**Published:** 2021-10-02

**Authors:** Rokeya Akter, Agnieszka Najda, Md. Habibur Rahman, Muddaser Shah, Sylwia Wesołowska, Syed Shams ul Hassan, Sidra Mubin, Parveen Bibi, Saeeda Saeeda

**Affiliations:** 1 Department of Pharmacy, Jagannath University, Dhaka 1100, Bangladesh; rokeyahabib94@gmail.com; 2 Department of Global Medical Science, Wonju College of Medicine, Yonsei University, Gangwon-do, Wonju 26426, Korea; 3 Department of Vegetable and Herbal Crops, University of Life Sciences in Lublin, 50A Doświadczalna Street, 20-280 Lublin, Poland; 4 Department of Pharmacy, Southeast University, Banani Street, Dhaka 1213, Bangladesh; 5 Department of Botany, Abdul Wali Khan University Mardan, Mardan 23200, Pakistan; parveentariq825@gmail.com (P.B.); syeeda177@gmail.com (S.S.); 6 Natural and Medical Sciences Research Center, University of Nizwa, Nizwa 616, Oman; 7 Institute of Soil Science and Environment Shaping, University of Life Sciences in Lublin, 7 Leszczyńskiego Street, 20-069 Lublin, Poland; sylwia.wesolowska@up.lublin.pl; 8 Shanghai Key Laboratory for Molecular Engineering of Chiral Drugs, School of Pharmacy, Shanghai JiaoTong University, Shanghai 200240, China; shams1327@yahoo.com; 9 Department of Botany, Hazara University Mansehra, Mansehra 21310, Pakistan; shahhu123@gmail.com

**Keywords:** cancer, radiotherapy, therapeutic, natural products, chemotherapy

## Abstract

Cancer is the second leading cause of death in the world. Chemotherapy and radiotherapy (RT) are the common cancer treatments. In addition to these limitations, the development of adverse effects from chemotherapy and RT reduces the quality of life for cancer patients. Cellular radiosensitivity, or the ability to resist and overcome cell damage caused by ionizing radiation (IR), is directly related to cancer cells’ response to RT. Therefore, radiobiological research is emphasizing chemical compounds ’radiosensitization of cancer cells so that they are more reactive in the IR spectrum. Recent years researchers have seen an increase in interest in natural products that have antitumor effects with minimal side effects. Natural products, on the other hand, are easy to recover and therefore less expensive. There have been several scientific studies done based on these compounds that have tested their ability in vitro and in vivo to induce tumor radiosensitization. The role of natural products in RT, as well as their usefulness and potential applications, is the goal of this current review.

## 1. Introduction

Cancer is a serious life-limiting disease. Many factors such as lifestyle, genetic variation, infection with viruses, and chronic inflammatory effects can affect cancer susceptibility. In recent decades malignant tumors were both better diagnosed and treated. Molecular-based care and conventional therapies like chemotherapy and radiotherapy are a positive development in cancer therapy [1,2]. The multifaceted complexity and diversity of tumors, the refractive complexity of conventional chemotherapy, and their adverse effects are still the first issue of this challenge: advancement of therapeutic therapies taking into account not just the particular tumor subtype, but also the patient’s genomic characteristics. The personalized therapies included chemotherapy, chemical therapy, immunotherapy, and radiotherapy (RT) [3]. Although traditional therapeutic therapies can have detrimental effects on the normal tissues too, the main goal of conventional radiation therapy is to give a regulated radiant exposure to a given tumor bulk and to affect carcinoma cells specifically with a high- or low-energy photon beam. In contrast to chemotherapy, which has experienced a continuing development of brand new drugs, the RT concept is the same for over one hundred years, with progress mainly affecting technology in that clinical field [3]. In fact, by imaging techniques combined with RT the dose can be delivered more accurately to its intend. However, treatment plans are generally the same for all tumors, regardless of their molecular profile, which plays a crucial role in the RT response [4]. At the present time, different types of RT neoplasms, including breast, ovarian, head/neck, lung, prostate, and lymphoma, have been treated [5]. There will be a direct or indirect exposure to radiation. The most critical aspect of RT is expected to be reactive oxygen species (ROS) formation due to RT. ROS plays an important role, contributes to death, and affects human cells in cancer cell exposure. The radiosensitivity is characterized as the vulnerability of cells to damaging ionizing irradiation effects, and cells with high rates of proliferation appear to suffer IR damage [6]. The biological impact on the irradiated tumor is mainly essential for cell radiosensitivity and is different from the tissue, which may create a difference between a reacting target and the non-response aspires. Radiosensitization plays a vital role in this, as a neoadjuvant for RTs, and chemicals that can sensitize cells of cancer have been used to improve treatment efficacy. In clinical practice, synthetic sensitizers are common and can be summarily classified as hypoxic and non-hypoxic based on their restore physiological intratumoral oxygen, which significantly decreases within the tumor bulk. Oxygen is permanently able, based on a oxygen fixation hypothesis, to stabilize radical damages to deoxyribonucleic acid (DNA) by radiation [7]. The ratio of the hypoxia/air radiation dose effect or ratio therefore describes the effect of IR in relation to the occurrence of oxygen. Nitroimidazole, misonidazole, etanidazole, and nimorazol are the most common hypoxic sensitizer. The nitro-group reduction reacts with the radicals of IR-DNA in the absence of oxygen, which stabilizes them in accordance with the hypothesis of oxygen fixation. This stabilization leads to a breakdown in the DNA spectrum and hence has effects on target hypoxic cells [8,9]. In recent years, the researchers have focused on the use of natural products as a coadjuvant for cancer treatment. Plants, bacteria, fungi, insects, spiders, marine organisms, and higher-order animals make up a large and diverse group of natural products. Natural products can be stored easily and are less costly than synthetic drugs. However, they reduce the adverse effects that worsen the often low quality of life of oncologic patients, along with the side effects of chemotherapy. An extensive analysis of the positive effects of natural products in combination with chemotherapy was conducted, however little information is known about its role of radiosensitization. Natural dietary supplements containing some ingredients such as Celastrol and curcumin promote the recovery from severe illness, and relieve chemotherapy and radiotherapy-induced side effects [10]. That’s why the review aims at covering in vitro, preclinical, and clinical state-of-the-art literature for certain natural products in the sense of RT and to explain how they affect IR response to cancer cells. Contrary to recent chemotherapy, which may interfere with tumor targets, RT is less dependent on the biological features of cancer being treated. In fact, each cancer has distinct characteristics linked to a different RT response and repetition after RT. The synergistic effects of radio-sensitizer compounds, recently introduced into clinical practice as a neoadjuvant for RT, may result in an increase in treatment response. However, the collateral effects of synthetic radiosensitizer aggravate those already created by RT. For this reason, several scientific projects are concerned with using natural products that can counteract RT tumor resistance mechanisms but still have less collateral effects. Our review focuses on providing an overview of the potential course of adoption of natural products in RT as an adjuvant and gives some insights (Figure 1).

## 2. Resveratrol

The exact mechanism of Resveratrol (RV) anti-proliferative effects is still being investigated, despite several in vitro cancer studies showing that resveratrol inhibits and suppresses tumor growth. Multiple signaling pathways are disrupted in malignant cells, resulting in uncontrolled cell proliferation, inhibited programmed cell death, and enhanced angiogenesis and uncontrolled cell migration [11]. It has been shown in the literature that resveratrol acts on cancer cells in multiple ways, including proapoptotic, antiproliferative, and anti-angiogenesis mechanisms, to name a few. TANK-binding kinase 1 (TBK1), for example, may be one of RVs direct targets [12]. The first indication of white hellebores was polyphenol RV isolated in 1940. RV has since been found in various sources of food, including red wine, raisins, mulberries, and peanuts [13,14,15]. RV is a natural polyphenol phytoalexin found in many crops or fruits normally eaten by human beings. The plant development has a function to defend against mechanical damage and invasion by harmful microorganisms including bacteria and fungi. In the last decades, beneficial effects from RV use, following a 1992 study by Renaud and De Lorgeril, which was also called the “French Paradox”, were thoroughly investigated. The study revealed that moderate red wine use was linked to coronary cardiac disease protection [16]. In combination with cardio protection, anti-aging effects and RV prevention have since been discussed [17,18]. In fact, while cardioprotection, aging, and other effects can easily be converted to the property of an “antioxidant”, one can be more dependent upon the “pro-oxidant” properties of the anti-cancer. The idea of hormesis is easily explainable because the same compound may have different activities that depend heavily on the dosage given, namely, the Swiss doctor Paracelsus, “The dose produces the poison”, and RV, which has two different activities depending on its concentration [19]. RV has proven to be a negative factor in the regulation of a wide variety of mechanisms, including cell growth and cell division [20]. RV treatment with 20 μM increases IR in non-small cell lung cancer at μ-rays of 0 to 8 Gy. The development of ROS and DNA in NSCLC cells is attributed to increased doubling-beach breaks in melanoma, which results in accelerated sinescene and cell death [21]. Increased in-vitro colony capacity for cancer cells development and increased DNA damage in spheroid cell culture in relation to the radiocensification of RV in IUdr alone cells resulted in combined cells with RV-20 μM and IUdR (iUdR) 1 icon and 2Gys radiation of γ. In a prostate cancer xenograft mouse study, the combination of RV has significantly hindered the growth of the tumor [22]. Additionally, the use of RV decreased tuber and weight in the nasopharyngeal carcinoma model, by 50 mg/kg/day (4 Gy/day) and radionuctible for a successive three-day period in connection with the treatment once IR or RV alone has been performed [23]. Recently, the radiosensory effects of RV have also been reported in breast cancer. Combination of RV-effects in the S-process phase in the human breast-cancer line (MCF-7), at 0, 10, 30, and 100 μM concentrations at 1, 2, and 3 Gy dose photon radiations caused cytototoxic symptoms and diminished cell proliferation. Interestingly, the results did not depend on the dosage of RV used, but instead on the mean irradiation concentration of 10 μM and 3 Gy [24]. In short, high doses of chronic RV were well tolerated and emphasized their function as an additional potential agent for cancer treatment [25].

## 3. Curcumin

Curcumin suppresses the signal transducer and activator of transcription 3 (STAT3) and nuclear factor kappa B (NF-κB) signaling pathways, both of which play important roles in the genesis and progression of cancer, as previously stated [26]. In prostate cancer cell lines and clinical samples, constitutive activation of the STAT3 and NF-B signaling pathways has been demonstrated [27,28]. In CL-5 xenograft tumors, curcumin has also been shown to promote apoptosis and cause down-regulation of epidermal growth factor receptor (EGFR), protein kinase B (Akt), and cMET cyclin D1 [29,30]. Curcumin has been shown to inhibit cell proliferation, cell cycle arrest, and stimulate apoptosis by modulating other transcription factors like activator protein 1 (AP-1), early growth response protein 1 (Erg-1), p53, -catenin, Notch-1, hypoxia-inducible factor 1 (HIF-1), and peroxisome proliferator-activated receptor alpha (PPAR-α) [31]. Curcumin is a promising compound for the treatment of cancer, a rotary polyphenolic agent [2,32]. Curcumin has been in Chinese and Hindu medicines for thousands of years, but curcumin has been an important attractor in recent decades because of its anti-cancer effect. The positive impacts of curcumin are antioxidant, anti-inflammatory, anti-proliferative, and anti-angiogenic [27,33,34]. In specific tumor cell lines and xenograft models, various curcumin experiments have been demonstrated as anticarcinogenic and therapeutic activity. Curcumin is well known for its efficacy in various models of animal cancer, including colon, breast, pancreas, lung, kidney and blades, blood, and skin [35]. Curcumin has a strong ability to selectively destroy cancer cells, without necessarily being harmful to non-malignant cells, as a cancer-preventative candidate [36]. Wide-ranging toxicological examinations and preclinical studies have shown that Curcumin is not difficult for mice, rabbits, dogs, and monkeys [37]. Even high doses (8–12 g/d) for several months in Phase II and Phase I clinical studies have demonstrated curcumin safety [37,38,39,40]. Pharmaceutical, metabolites, and systemic bio-disposability have shown insufficient intake, fast metabolism and limited systemic biodisposability for rodents and humans [41,42]. Interestingly, curcumin is an important agent in many forms of cancer during animal experiments despite its limited bioavailability. It is not clear if the effectiveness is due to the unexplained effects of curcumin. Five patients received three treatments a day in another study at Cleveland Clinic in Florida, with a combination of curcumin and quercetin, for an average time of six mos. In all instances, in accordance with the particular values the number and scale of polyps are reduced [43]. The findings revealed that the number of aberrant crypt foci (ACF)with curcumin is marginally lower at 4 g, which indicates the existence of early pre-invasive lesions may cause curcumin carcinogenicity. However, the remaining ACF dispute in the context of colon cancer biomarkers, nonrandomization and placebo group interpretations of the study was limited [44]. In a Phase II clinical trial for patients with chronic diseases, curcumin-effectiveness in the treatment of human pancreatic cancer was reported. After two seconds of progression, patients receive 8 g of curcumin per mouth daily. A clinical Phase 2 trial shows that gemcitabine and curcumin are mixed in patients with pancreatic cancer [45]. Bayet-Robert et al. were seeking advanced and metastatic curcumin and docetaxel combinations in 14 patients. This study shows that vascular endothelial growth factor (VEGF) levels have been reduced and that combined therapy has been successful. Hopefully, further data will soon be available to prove curcumin’s anti-cancer effects, especially measures to verify the in vivo molecular goals based on the mechanisms [46]. Curcumin treatment reduces the levels of free radicals and MDA-DNA adduct in rat model [47]. In patients with various types of malignancy, chemo- and radiotherapy of 500 mg, lecithinized delivery system of curcumin alleviates the burden of side effects [48].

## 4. Vitamin D

Vitamin D is known to have a wide range of bioactivities, including cancer, linked to various clinical conditions. Besides its role in the homeostasis of calcium and bone metabolism [49]. Vitamin D2 is mainly produced by yeast or irradiation of ergosterol [50,51]. The binding of the Vitamin D Receptor is used to mediate the bulk of the 1, 25-(OH) 2D3 anti-cancerous activity. The 1,25-(OH)2D3 cells bind to the vitamin D receptor (VDR) and the retinoid X receiver in the cell nuclear is heterodimerizes [52]. This hederodimere binds the reaction portion of vitamin D in the target genes and stimulates the regulation of many genes including cell growth maintenance, differentiation, and apoptosis and inflammation [53,54,55]. A growing number of laboratory experiments in vitro and in animals have shown good anti-tumor efficacy for vitamin D and closely investigated mechanisms in cells and molecules [56,57]. It is seen that vitamin D use together with radiotherapy can have a positive effect on cancer treatment [58]. While comprehensive studies have been performed to reverse the link between vitamin D and cancer risk, the disease data available has been unreliable until now. Exceptional for populations in areas with low UV exposure is the recorded increase in the prevalence of several cancers including prostate, colon, and breast [59,60,61,62,63,64]. Many adverse symptoms, including nausea and vomiting, fatigue, exhaustion, lethargies, and agitation, such as hyperphosphatemia and hypercalciuria, have been associated with the insufficient consumption of vitamin D. The net effect is toxicity if the daily intake is greater than 10,000 vitamin D IU regularly [65,66]. Many analogs of vitamin D were outlined in order to reduce these side effects [56,67]. In addition, recent findings have studied intermediate calcitriol administration at exceptionally high doses that only lead to intermittent, antiproliferative hypercalcemia [68,69]. The optimum dosage, the ideal biological dosage, and the best pacing for the available formulations of vitamin D are still unanswered. Vitamin D and its metabolite, as well Como analog medicines have been used for the prevention and treatment of various cancers, particularly for prostate, breast, and colorectal cancer in a large number of human intervention trials.

## 5. Celastrol

Celastrol is an anti-inflammatory vitamin extracted from *Tripterygium Wilfordii*’s thunder wine, commonly used as a treatment for much pathology in conventional Chinese medicine and is renowned for its non-inflammatory impact. Celastrol has been a successful choice for further study into cancer biology by finding its inhibitory proteasomic activity and anti-metastatic ability [70]. Celastrol has recently been demonstrated to effectively decrease tumor growth, migration, and angiogenesis in a variety of tumor models, both in vitro and in vivo 18–20. Celastrol reduces the CIP2A/c-MYC signaling pathway and inhibits proliferation, migration, and invasion [71]. Celastrol also stops ovarian cancer cells from migrating and invading by inhibiting nuclear factor kappa B (NF-κB) pathway [72]. Celastrol also affects the expression of a number of oncogenes and tumor-suppressor genes, such as CXCR4, the VGEF receptor, and CIP2A. (the p90 tumor-associated antigen) [73]. In 0.4 μM, not 0.2 μM, the dose-dependent IR-induced cytototoxicity in cell and clonogenic cell killing demonstrated a substantial rise in Celastrol. Radiation changes are also attributed to the interaction with radiation-caused DNA damage repair cycle. Following radiation damage induced, the kinetics of appearance and disappearance of a marker (αH2AX), were then monitored through immunofluorescence and Western blotting testing. The analysis reveals, while cells have long been irradiated, that the cell in the célastrolium treated with celastrol in combination with IR has been positively μH2AX. In cells undergoing combined celastrol and IR treatment, however, apoptosis markers were more common than in cells treatment with X-rays. A PC-3 xenograft in athymic NCr-nu/nu maus has tested the effect of Celastrol or in vivo IR. Celastrol was well absorbed and was able to prevent the tumor duplication in combination with IR alone. In fact, the relation between celastrol and exposure to radiation greatly improved apoptosis and decreased the blood vessel by histology. Celas are linked to the γ-irradiation of the human lung cancer cell line of the NCI-H460. The radiation dose was expected to influence cell growth and survival and was investigated following celastrol therapy to demonstrate radiation sensitive targets such as EGFR, ErbB2, Survivin, and Akt. The resulting disruption of the proteins in conjunction with HSP90 celastrol-dependent significantly reduced all other marker values with the exception of Akt [74]. Celastrol also has shown to depend on its quinone methide motion, which improved the ROS after IR production for its radiosensitizing influence in lung cancers cells [75]. The clonogenic test indicates that Celastrol + IR therapy decreases the survival of the two cell lines and in vivo tests the IR reaction by using Celastrol. The pre-clinical model was a lung tumor model that was used for A549 cell line during 12 days of celastrol and IR (10 Gy) combination therapy. Days 6 and 12 saw the slaughter of mice and the testing of H&E tumors. The study shows that intratumoral necrotics in combination nutritional tumors was greater than in mice treated with Celastrol or IR alone [76].

## 6. Zerumbone

Zingiber (ZER) Smith cytotoxic compound is an isolation part of *Zingiber zerumbet* [22,77]. It is used as a condiment for food and medicine in eastern countries for its phytomedical properties from ancient times [78]. The proliferation and anti-tumor properties of various tube types such as the breast, pancreas, colon, lung, and skin were also shown to be anti-inflamative [79,80,81]. Indeed, in recent years a number of studies have shown that Zerumbone influences cancer sensitizing during IR therapy, including IR and cell cycle repair and apoptotic pathway function [82,83]. Regularly, some researchers have described the combined therapy in NCI-H1299 cell line 48–72 h after ZER (10 μg/mL) and β-ray (range from 5–10 Gy) irradiation effects of the Zerumbone. In addition, before the treatment of PC3 and DU145, cell life was decreased until reaching different doses of IR (0–6 Gy), μ-H2AX was removed and the expression of ataxia telangiectasia mutated (ATM), Janus kinase 2 (JAK2) gene, and STAT3 phosphorylated proteins, all involved in DNA damage preparation (10 μM) until human prostate ZER cell treatments, were decreased [84]. Brain tumors are the leading cause of cancer-related death in children [85]. The incidence of primary malignant brain tumors is increasing, of which 80% consist of high-grade malignant tumors such as glioblastoma multiform (GBM) [86]. Another study has reported that treatment with Zerumbone suppressed FOXO1 and Akt phosphorylation due to inactivation of IκB kinase α (IKKα) while activating caspase-3 protein and Poly (ADP-ribose) polymerase (PARP), which resulted in decreased cell viability, and induction of apoptosis in GBM cells [87].

## 7. Ursolic Acid

The family of triterpenoids belongs to Ursolic acid (UA), including the above-mentioned celastrol. This is found in the skin of many vegetables, including strawberries, blueberries and plums, and in many herbs such as rosemary and thyme. While the use of natural molecules has been unaware for centuries of the pharmacological effects of UA, which has anticancer, anti-inflammatory, and anti-microbial activity, it has recently been demonstrated [88]. Its application has also been recently emphasized for radiosensitization. A notable decrease in cell viability relative to untreated CCs was seen in the DU145 human prostatic cell line in 30 μM UA 24 h before Gy-irradiance (5 Gy). As a result, cells and compact or broken nuclides, caspase-3 amplification, cleaved PARP and DNA were decreased. Cell viability was reduced, Apoptotic waterfall Activation and an elevated amount of ROS were also observed in human colon carcinoma CT 26, and mouse melanoma cells B16F10 treated all under same conditions as DU145 cells. Mouse implanted in B16F10 cells has been blocked for 2 weeks and treated with 100 mg/kg and 4 Gy IR via the down regulation of Bcl-2, Survivin via the tumor test Western blot [89]. After UV treatment to human or cancer cells, UA therapy caused a differential operation. The human cell line CRL-4000hTERT-Rpe and CRL-11147 melanoma cells of skin were both treed with 1 μg/mL UA in an assessment of differential ROS-mediated UV production, cell stoppage, and mortality at least 8 h before UV radiation. However, clonogenic treatment and the expression of YO-PRO-1 has been checked for therapy with UA, with the aim precisely of potentiating apoptosis that can induce optical radiation and cell death in skin melanoma cells rather than in RPE cells [90]. NSCLC cells and, in particular, HIF-1α-expressing cells were intrigued by the findings when they were irradiated with UA after pre-irradiation relative to other cell lines. These sensitizations have been linked to increased DNA damage rates as one of the most effective ROS scavengers, measured by a study of the formation of micronuclei, which have dramatically reduced endogenous glutathione levels [91]. Acute irradiation-induced deficiencies in contextual learning and memory, as well as novel object recognition memory, were found to be improved by UA. In the subgranular zone, however, the therapy worsened the radiation-induced loss in neurogenesis. An increase in mitochondrial dysfunction caused by domoic acid in mice has been demonstrated to be improved by UA through modulating the signaling pathways for Forkhead box protein O1 (FoxO1) and PI3K/Akt [92]. There was additional evidence that D-galactose caused neurodegenerative alterations might be treated with UA through antioxidant and anti-inflammatory pathways. Apart from better performance in the step-through test and Morris water maze, therapy with UA was demonstrated to decrease advanced glycation end products (AGEs), receptor for AGE, ROS, and protein carbonyl in the prefrontal cortex [93].

## 8. Withaferin A

Withaferin A (WA) is a steroid of the lactone of a major category of natural steroids known as mitanolides. The result was an extract of the wild plant leaves *Withania Somnifera*, also known as *Ashwagandha* or *Winter Cherry*, from the 1950s. Work on the antitumor activity in WA began immediately after isolation and demonstrated the effects of WA on nasopharyngeal and osteosarcoma cell carcinomas [94,95]. Several experiments showed since that time, that WA is both in vitro and in vivo a natural anticancer agent [96]. As forecast, WA and a single RT have shown an inhibition of tumor growth and tumor-free survival and improved memory specificity training. Mice treated every 8 days at 5 mg/kg have attained 40 percent tumor-free survival, with the average survival time of 120 days rising to 100 percent free tumor, at a cumulative dose of 30 mg kg per second. In WA 5, 7, or 10 days following inoculation similar results were obtained indicating that the tumor growth effects of WA can partly be solved. Treatment for WA and RT was unsuccessful in advanced tumor stages. In general, treatment with RT alone cannot cause positive effects especially in mice [97]. Before the individual 30 Gy dosage irradiation and multiple tumor response parameters were measured, the mouse was treated with incremental WA dose of 10 to 60 mg/kg. Nonetheless, in 45% of cases with 40 to 60 mg/kg of mice, complete remission was completely convincing at 55% and partial remission [98]. The results of WA + RT in fibrosarcoma were studied and melanoma symptoms tested on the same laboratory conditions. The findings were roughly the same as expected [99]. Over the past years the emphasis on withaferin A’s radiosensitizing impact has also been on the mechanisms that are compromised following the WA therapy. One of the in vitro study reported that WA reduced the viability of the human histiocytic cell line U937 [100]. Most experiments combine the 0.5 μM subtoxic dosage; however, with the 10 Gy radiation as the wafer, cytoplasmic accumulation and nuclear condensation will effectively induce around 40% cell death as well as other morphologic changes in the apoptosis, e.g., cell shrinking. In addition, the IR-accompanied administration of WA leads to higher ROS output, increased PARP expression, decreased Bcl-2 activation of JNK and p38 signals known to be triggered by further cellular voltage, like ROS [101]. Same group of researchers have been derived from the Withaferin A vaccine 4 μM and 10 Gy from the X-ray cells vaccine in caki (renal carcinoma), SC-Hep1 (liver carcinoma), MDA-MB231 (width cancer), and HeLa (cervical cancer) cells in other lines of cells [102]. According to a study by Widodo et al., WFA selectively activated p53 in tumor cells treated with Ashwagandha leaf extract, leading to growth arrest and apoptosis [103]. In addition to other pathways, WFA-induced apoptosis has been widely documented. ROS are generated when mitochondrial respiration is inhibited by WFA, according to research by Hahm et al. As compared to normal human mammary epithelial cells (HMEC), MDA-MB-231 and MCF-7 cells produced more ROS after treatment [104]. It has been shown that WFA treatment induces apoptosis in breast cancer by altering mitochondrial dynamics [105].

## 9. Emodin

Emodin is a natural phenol agent derived from roots and rhizomes of several species, including the *Cascara sweetheart* and the *Cascara palmatum* Chinese herbs [106,107]. Emodin is a similar, endogenous ROS generator with electron transfer capability to DMNQ (2,3-dimethoxy-1,4-naphtoquinone) and mitochondrial ubiquinone [108]. It works against bacteria, antiviral products, inflammatory diseases, and cancer [109,110]. The methods used to inhibit cancer formation in Emodin remain unknown, while leukemia, breast cancer, colon cancer, and lung cancer, have been shown to have an effect against tumors [111]. In many cancer cell lines, important findings have also been found. The different doses of HeLa cervical cancer cell lines induced a change in some radiobiological parameters in the survival curve before being exposed to different dose of radiation (0, 2, 4, 6, 8, 10 Gy) at various doses of the Emodin-alone (0.5, 100 and 200 μM) dose. In the clinical practice (SF2), the average fractional dose of 2 Gy and concentration-dependent increase in sensitivity ratios SER (D0) and SERDq were reduced overall to the medium lethal dose (D0), quasi-threshold dose (Dq), and extrapolation dose (N). The distribution of cells and apoptosis studied showed an increased number of G2/M and sub-G1 cells within 24, 48, and 72 h after 50 μM AE and 4 Gy IR treatments. This combined treatment also increases Cyclin B, γ-H2AX, and ALP expression [112]. Also in the same therapeutic method, p53 mutant (Mut) murine cell sarcoma was employed. Nuclear survivors exposed to 50 μM AE before 2 Gy X-rays radiation and decrease of the nuclear transportation protein, called chromosome region maintenance 1 survivors, export from the nucleus to cytoplasm [113]. Emodin increased the cytotoxicity generated by gefitinib in two non-small cell lung cancer (NSCLC) cell lines, A549 and H1650, according to Chen et al. Emodin improved a gefitinib-induced drop in phospho-ERK1/2 and Rad51 protein levels by increasing Rad51 protein instability at low dosages of 2–10 M [114]. By activating a ROS-activated ATM-p53-Bax signaling pathway, Lai et al. found that Emodin promoted mitochondria-dependent apoptotic cell death in human lung adenocarcinoma A549 cells. The proteins ERCC1 and Rad51 are required for nucleotide excision repair and homologous recombination [115]. Platinum-containing drugs such as cisplatin or carboplatin are the most significant chemotherapy treatments for patients with advanced NSCLC. Resistance to platinum-based medications is one of the most significant hurdles to cancer treatment, and it is frequently linked to a poor prognosis in NSCLC patients. In human NSCLC cell lines, Emodin was found to boost the cytotoxicity caused by cisplatin in a synergistic manner [116].

## 10. Berberine

Berberine(BBR), a part of the alkaloid derived from many medicinal plants, including *Huang Lian*, has low toxicity. It is also commonly used in China as a medication for gastrointestinal pain and has been tested for diabetes mellitus type 2 and hypercholesterolemia in clinical studies [117,118]. Research has shown that BBR has a variety of cancer cells antitumor activity [119,120,121]. The progression of the cell cycle and the promotion of apoptosis are frequently inhibited. A study found that BBR has radiosensitization in cells that cause lung cancer [122]. A follow-up study showed that BBR significantly radiosensitizers esophageal cellular cancer (ESCC) at low levels. In cell lines (KYSE30; KyS450, KYSE410, EC109; TE-1), BBB (15 μM) was tested for 24 h with X-radiography (2–6 Gy) susceptibility to radiation was important. The downregulation of RAD51 in DSB repair, as experimental data demonstrated, has mediated this effect. The ESCC human tissue over-expression of RAD51 suggested this protein may be employed as a radiation reaction biomarker. Indeed, in non-malignant cells at radiosensitization stages, BBRhas not determined any influence or down-regulation of RAD51. There is therefore an expected radiosensitization effect of Berberine unique to the cells of ESCC [123]. One cell of a human prostate cancer (PC-3) line had a high apoptotic rate of γ-irradiation (4–6 Gy) with berberine (30 μM) for 24 h. The apoptosis process aimed at improving the ROS of this receptor for prostate cancer. In addition, the combined action of BBR on prostatic cancer cells and mechatribes such as Bcl-2 NF-kB-p53, P38 and JNK radiosensitizing and expanding has shown that a range of molecules involved in apoptotic, cell cycle, and radiation expression are deregulated [124,125,126,127]. Finally, BBR’s role in radiosensitization was tested in models for breast cancer. BBR (15 μM) was treated with a variable dose of X-ray (1–4 Gy) in the cells of breast cancer, MCF-7 and MDA-MB468. The findings indicate that cell cycle retention, mechanisms for restoration of μH2Ax focus-inhibited DSBs, and down-regulation of RAD51 are followed by a BBR therapy [128]. Immunotherapy for the treatment of cancers has gotten a lot of interest recently. BBR has been found to have anti-tumor immunotherapy properties. In a study, BBR inhibited the release of IFN-γ, TNF-α, interleukin (IL)-6, and IL-1 from LPS-stimulated lymphocytes by acting as a dopamine D1- and D2-like receptor antagonist [129]. BBR also reduced TNF-α and IL-1 levels and inhibited CD4+ T cell proliferation, which helped to alleviate autoimmune neuropathy [130]. Furthermore, BBR blocked STAT1 phosphorylation, resulting in IFN-γ induced IDO1 expression suppression. These findings suggested that BBR could be a promising therapeutic target for tumor immunotherapy [131].

## 11. Selenium

Selenium (Se), which is naturally found in the form of two inorganic compounds, selene and selenate, is an important ingredient for humans, plants, and micro-commonwealth as well as organic derivatives. Sodium selenite, usually associated with an antioxidant activity, is an oxidant that helps cells to be more prone to oxidative stress in spite of the other selenium compounds. Several experiments suggest that its cytotoxic effects are more vulnerable to phagocytic cell activity and apoptotic pathways due to the overt or indirect activation of the natural killer cells (NK) and the induction of disulfide exchanges on the surface of cancer cell membranes [132,133]. Therefore, as described by numerous studies, the use of selenite appears to have promising anti-cancer effects, including with RT. In A375, human melanoma cells also radiosensitizing effects of Se were found. Liua et al., in particular, investigated the effects combined with bevacizumab and X-rays of a highly hemocompatible, membranously covered ultrasmall selenium nanosystem (2–8 Gy). After combined treatment (17.5%), data from the test showed a growth of caspase-mediated apoptotic pathways within the A375 cell area. Increased A375 cell proportions in the activated cleave caspases 3/8/9 and PARP cleavage alone (56.2%) in RBCs or RBCs@Se/Av alone (96%). Moreover, this procedure leads to improved development of ROS, mitochondrial ROS fragments and multiple DNA damage marker levels, while also reducing expressiveness of VEGF and VEGF2 [134]. Despite several investigations on the pharmacodynamics (PD) of Se in normal and malignant cells, it is still unknown which form and dose of Se may be administered safely and has the best differential effect in normal and malignant tissues, particularly when combined with chemotherapy and radiation. Although the pharmacokinetic (PK)-PD link has not been demonstrated in people, current Se doses are empirical or guided by PK. As a result, the best form and dose of Se to employ with chemotherapy or radiotherapy is unknown. To the contrary, Joel et al. have shown that human white blood cells (WBC) can be used to quantify PD biomarkers of Se effects, which will allow clinical research to examine Se PD/PK in order to establish the appropriate Se drug and dose to be put into potentially pivotal trials [135].

## 12. Genistein

Genistein (SOY ISA) prevents the spread of the cell and thus improves apoptosis by inhibiting tyrosine activity and DNA topoisomerase protein kinases 2. These molecules also help the mechanism of DNA reparation and anti-angiogenic and anti-tumor activity [136,137]. In several studies, Genistein in vitro has shown that it inhibits cancer cell growth, such as lymphoma and melanoma [138]. Experimental results have shown that Genistein (40 μmol/L) treatments and I-radiation (4 Gy) are combined, which significantly inhibit cervix cellular cancer (Hela) growth and increase radiosensitivity down-regulation [139]. This receptor has been absent from usual isolated tissues and malignant tumors have been extensively exposed [140]. Mortality levels were linked to decreased mortality and increasing recurrence and clinical resistance; Genistein has therefore been recommended to reduce the dose of IR and possible RT adverse events [141]. Based on earlier work demonstrating Genistein’s capacity to suppress cell growth of cervical tumors, Yashar et al. assessed the possible role of the compound as a radiosensitizer in other cervical epithelial cancer [142,143]. Experiments have shown that Genistein reduced cell damage caused by oxidative stress in the A549 cell line; it reduced ROS and the antioxidant component glutathione [144]. Genistein has an effect on the methylation status of DNA: researchers have found, in particular, that methylation inhibition in the Promoter1 region of Keap1 implied an increase in the gene transcription rate [145,146]. The result was nuclear factor erythroid 2-related factor 2 (Nrf2), which is an antioxidant factor and the oxidative deregulation of the system [147,148]. Apoptotic and A549 cell radiosensitivity is improved through this experiment. This mechanism includes an interesting pathway for Keap1 and Nrf2, in standardized MRC-5 cells in the lung fibroblasts. Apoptotic and A549 cell radiosensitivity is improved through this experiment. Of note, the Keap1/Nrf2pathway involves uniform MRC-5 cells with lung fibroblast [149]. This combination Genistein IR therapy led to a reduction in Bcl-X, which is a recognized influence in the treatment of lung cancer, as seen in some research [150]. Bcl-x also took part in molecular interactions with Beclin-1 protein modulation of autophagy [151,152]. In short, the authors suggest that Genistein may affect the radiosensitivity of NSCLC cells, as they can regulate Bcl-x cytoplasmic expression levels and therefore apoptotic and autophagic processes [153]. Different forms of cancer have been carefully examined to determine Genistein’s molecular mechanism of action. Angiogenesis, angiogenesis and metastasis are all modulated by genistein. In terms of its molecular targets, Genistein has caspases as well as the NF-κB, extracellular signal-regulated kinase 1/2 (ERK 1/2), mitogen-activated protein kinase (MAPK), and the Wingless and Integration 1/-catenin signaling pathway as well as phosphoinositide 3-kinase/Akt (PI3K/Akt) [154]. Genistein-induced stress and its downstream targets have also been found to trigger apoptosis in cancer cells, together with transcription factors [155].

## 13. Future Perspectives

We are widely aware that “one size fits all” is not used for cancer treatment because generic medical guidelines are incorrectly treatable for patients who do not offset the dynamical nature of cancer. The quest for the best cure for particular neoplasms is therefore one of science’s most challenging problems. Today, with the development of the sequencing techniques and the expression of genes, we are aware of the importance of increasingly customized treatments as tumors that affect the same organ can be divided further into subgroups with a certain biological profile, which prevents treatments benefiting si-tumors. Since decades of relentless cancer studies, more effective treatments to personalize treatment have been built in the light of both the disease and the patient to be treated. Scientific methods including chemotherapy and RT have been applied, although for the first time, new and more powerful drugs have been developed, and since the detection of radioactivity and its initial use in cancer, which took place in 1896, they have been based on the same principles [156]. RT can deliver a certain dose to the tumor directly in relation to chemical therapy, thereby limiting tissue damage. It is precision in the use of harden therapy to save healthy areas surrounding the tumor. Thanks to their existence the most energy charged particles including protons and carbon ions will deposit with little diffusion [157,158]. Both traditional RTs, using photons (gamma or X-rays), and harden therapy may cause cell death by altering the DNA’s target structure. DNA breaks may be directly induced if there are double beach helix effects or if there is an indirect definition of the effects of ROS production triggered by RT. Nearly every molecular structure in the cells can also be oxidized and killed, not only causing DNA damage [159]. However, cancer can also acquire RT resistance, as often happens with chemotherapy. Therefore, RT can be coadjusted by the application of radiosensitizing compounds. Several medications are used for this reason today that are generally referred to as hypoxic and nonhypoxic (e.g., nitroimidazoles and halogenated pyrimidines) radiosensitive agents, which may have widespread downstream consequences. Nutraceuticals, which can echo the effect of radiosensitizers with synthesis, may help solve this issue since their toxicity is small. The interest in natural compounds to treat a variety of pathologies has been increased lately not only due to their less toxic effects, but also due to their low cost. The benefits of natural compounds have long since been recognized for their health promotion, and their use in medical treatment is central to conventional medicinal products, including traditional Chinese and Ayurvedic medicinal products. The benefit of nutraceuticals has been the use of hypertension, diabetes, and osteoporosis and lipid control. They were used in clinical practice as a neoadjuvant to chemotherapy [160,161,162]. It cannot be concluded that nutraceuticals products also contribute to the mediation of radiation exposure. According to several scientific documents, it works as an anticircumcisant that demonstrates its positive effects as radiosensiblists, we are trying to collect data on natural materials such as turmeric, resveratrol, vitamin D, withaferin, celastrol, ursolic Acid, Zerumbone, emodin, berberine, Genistein, and selenium (Table 1). This is demonstrated by the general capacity of the cell to produce down-regulation BCL-2, PARP increases, and Caspa-3 cleavage. These are the most common biochemical findings of tumor radiosensitization. All results are based on the uniqueness of nutraceuticals. The nutraceuticals pathways such as cell migration, swelling, autophagy, and ROS production are summarized in Figure 2. The nutraceuticals pathways such as cell migration, swelling, autophagy, and ROS production are summarized in Figure 2. Many of the protective mechanisms behind the products of nutraceuticals still need clarification and description. Deeper understanding of the key pathways for radiosensitization of nutraceuticals can be a better way to function and can help recognize new cell-sensitization targets.

## 14. Concluding Remarks

A powerful and well-tolerated radioprotector for normal tissue is needed because RT is a mainstay of cancer treatment and patients often suffer from side effects as a result. ROS are the main dangers of irradiation. Many medicinal plants have been used in natural products for hundreds of years, indicating that they are well tolerated. But even though a complete radioprotection is not possible, the role of natural products as modulators of the cell cycle, DNA repair, and antioxidative stress reduction is becoming more and more evident. The goal of improving quality of life without compromising therapeutic efficacy requires further elucidation of the properties of natural products and the mechanisms by which they prevent the side effects of chemotherapeutic drugs and radiation, in order to aid in the rational combination of natural products with anticancer drugs to optimize cancer treatments.

## Figures and Tables

**Figure 1:** Some beverages containing natural products that show health-promoting and relieve chemotherapy and radiotherapy-induced side effects.

**Figure 2:** Different natural compounds treatment might affect the migration, inflammation, and autophagy and ROS cell pathways.

**Table 1:** Represents the effect of radiosensitizers on the most common natural compounds.

Natural Products	Chemical Structure	Target of Tumors	Types of Treatment	Mechanism of Action	References
Resveratrol		Breast Cancer, Glioblastoma, Head and Neck squamous Cancer, Melanoma, Nasopharyngeal	γ-rays X-rays	Help to cure breast cancer	[21,24,163]
Curcumin		Breast cancer, Colonrectal Cancer	γ-rays X-rays	Help to reduce colonrectal cancer and breast cancer	[164,165]
Vitamin D		Colon and breast cancer	-----	Help to cure colon cancer	[166,167]
Celastrol		Prostate Cancer	γ-rays X-rays	Help to cure c prostate cancer	[168]
Zerumbone		Glioblastoma, Colonrectal Cancer	γ-rays X-rays	Curecolonrectal cancer	[169,170]
Ursolic Acid		Gastric Cancer	γ-rays X-rays	Help to reduce gastric cancer	[171]
Withaferin A		Carcinoma	γ-rays X-rays	CureCarcinoa	[97]
Emodin		Carcinoma, cervical cancer	γ-rays X-rays	Help to reduce cervical cancer	[112]
Berberine		Prostate cancer, Human breast cancer	γ-rays X-rays	Help to reduce prostate cancer, human breast cancer	[128,172]
Selenium	Se	Cancer cells	γ-rays X-rays	Eliminate cancer cells	[132,133]
Genistein		Cervical Cancer	γ-rays X-rays	Help to reducecervical cancer	[142,153]

## Data Availability

Not Applicable.

## Abbreviation

ACF	Aberrant crypt foci
AGEs	Advanced glycation end products
Akt	Protein kinase B
AP-1	Activator protein 1
ATM	Ataxia telangiectasia mutated
DNA	Deoxyribonucleic acid
EGFR	Epidermal growth factor receptor
Erg-1	Early growth response protein 1
FoxO1	Forkhead box protein O1
GBM	Glioblastoma multiform
HIF-1	Hypoxia-inducible factor 1
HMEC	Human mammary epithelial cells
IKKα	IκB kinase α
IR	Ionizing radiation
JAK2	Janus kinase 2
MAPK	Mitogen activated protein kinase
NF-κB	Nuclear factor kappa B
NK	Natural killer cells
Nrf2	Nuclear factor erythroid 2-related factor 2
NSCLC	Non-small cell lung cancer
PD	Pharmacodynamic
PI3K	Phosphoinositide 3-kinase
PK	Pharmacokinetic
PPAR- α	Peroxisome proliferator-activated receptor alpha
ROS	Reactive oxygen species
RT	Radiotherapy
RV	Resveratrol
STAT3	Transducer and activator of transcription 3
TBK1	TANK-binding kinase 1
UA	Ursolic acid
VDR	Vitamin D receptor
VEGF	Vascular endothelial growth factor
WA	Withaferin A
WBC	White blood cells
ZER	Zingiber

## References

[1] Karthika C., Hari B., Rahman M.H., Akter R., Najda A., Albadrani G.M., Sayed A.A., Akhtar M.F., Abdel-Daim M.M. (2021). Pharmacotherapy, Multiple strategies with the synergistic approach for addressing colorectal cancer. Biomed. Pharmacother..

[2] Epstein J., Sanderson I.R., MacDonald T.T. (2010). Curcumin as a therapeutic agent: The evidence from in vitro, animal and human studies. Br. J. Nutr..

[3] Forte G.I., Minafra L., Bravatà V., Cammarata F.P., Lamia D., Pisciotta P., Cirrone G.A.P., Cuttone G., Gilardi M.C., Russo G. (2017). Radiogenomics: The utility in patient selection. Transl. Cancer Res..

[4] Bravatà V., Cava C., Minafra L., Cammarata F.P., Russo G., Gilardi M.C., Castiglioni I., Forte G.I. (2018). Radiation-induced gene expression changes in high and low grade breast cancer cell types. Int. J. Mol. Sci..

[5] Baskar R., Lee K.A., Yeo R., Yeoh K.-W. (2012). Cancer and radiation therapy: Current advances and future directions. Int. J. Med. Med. Sci..

[6] Calvaruso M., Pucci G., Musso R., Bravatà V., Cammarata F.P., Russo G., Forte G.I., Minafra L. (2019). Nutraceutical Compounds as Sensitizers for Cancer Treatment in Radiation Therapy. Int. J. Mol. Sci..

[7] Grimes D.R., Partridge M. (2015). A mechanistic investigation of the oxygen fixation hypothesis and oxygen enhancement ratio. Biomed. Phys. Eng. Express..

[8] Bonnet M., Hong C.R., Wong W.W., Liew L.P., Shome A., Wang J., Gu Y., Stevenson R.J., Qi W., Anderson R.F. (2018). Next-generation hypoxic cell radiosensitizers: Nitroimidazole alkylsulfonamides. J. Med. Chem..

[9] Rauth A. (1984). Pharmacology and toxicology of sensitizers: Mechanism studies. Int. J. Radiat. Oncol. Biol. Phys..

[10] Zhang Q.-Y., Wang F.-X., Jia K.-K., Kong L.-D.J.F. (2018). Natural product interventions for chemotherapy and radiotherapy-induced side effects. Front. Pharmacol..

[11] Tagde P., Tagde P., Tagde S., Bhattacharya T., Garg V., Akter R., Rahman M.H., Najda A., Albadrani G.M., Sayed A.A.J. (2021). Natural bioactive molecules: An alternative approach to the treatment and control of glioblastoma multiforme. Biomed. Pharmacother..

[12] Youn H.S., Lee J.Y., Fitzgerald K.A., Young H.A., Akira S., Hwang D.H. (2005). Specific inhibition of MyD88-independent signaling pathways of TLR3 and TLR4 by resveratrol: Molecular targets are TBK1 and RIP1 in TRIF complex. J. Immunol..

[13] Signorelli P., Ghidoni R. (2005). Resveratrol as an anticancer nutrient: Molecular basis, open questions and promises. J. Nutr. Biochem..

[14] Shankar S., Singh G., Srivastava R.K. (2007). Chemoprevention by resveratrol: Molecular mechanisms and therapeutic potential. Front. Biosci..

[15] Rahman M.H., Akter R., Behl T., Chowdhury M.A., Mohammed M., Bulbul I.J., Elshenawy S.E., Kamal M.A. (2020). COVID-19 outbreak and emerging management through pharmaceutical therapeutic strategy. Curr. Pharm. Des..

[16] Renaud S.D., de Lorgeril M. (1992). Wine, alcohol, platelets, and the French paradox for coronary heart disease. Lancet.

[17] Ko J.-H., Sethi G., Um J.-Y., Shanmugam M.K., Arfuso F., Kumar A.P., Bishayee A., Ahn K.S. (2017). The role of resveratrol in cancer therapy. Int. J. Mol. Sci..

[18] Li J., Zhang C.-X., Liu Y.-M., Chen K.-L., Chen G. (2017). A comparative study of anti-aging properties and mechanism: Resveratrol and caloric restriction. Oncotarget.

[19] Rahman M.H., Akter R., Bhattacharya T., Abdel-Daim M.M., Alkahtani S., Arafah M.W., Al-Johani N.S., Alhoshani N.M., Alkeraishan N., Alhenaky A.J. (2020). Resveratrol and Neuroprotection: Impact and its Therapeutic Potential in Alzheimer’s disease. Front. Pharmacol..

[20] Rahman M., Rahman M., Hossain M., Biswas P., Islam R., Uddin M.J., Rhim H.J. (2020). Molecular insights into the multifunctional role of natural compounds: Autophagy modulation and cancer prevention. Biomedicines.

[21] Luo H., Yang A., Schulte B.A., Wargovich M.J., Wang G.Y. (2013). Resveratrol induces premature senescence in lung cancer cells via ROS-mediated DNA damage. PLoS ONE.

[22] Chen Y.-A., Lien H.-M., Kao M.-C., Lo U.-G., Lin L.-C., Lin C.-J., Chang S.-J., Chen C.-C., Hsieh J.-T., Lin H. (2017). Sensitization of radioresistant prostate cancer cells by resveratrol isolated from arachis hypogaea stems. PLoS ONE.

[23] Tan Y., Wei X., Zhang W., Wang X., Wang K., Du B., Xiao J. (2017). Resveratrol enhances the radiosensitivity of nasopharyngeal carcinoma cells by downregulating E2F1. Oncol. Rep..

[24] da Costa Araldi I.C., Bordin F.P.R., Cadoná F.C., Barbisan F., Azzolin V.F., Teixeira C.F., Baumhardt T., da Cruz I.B.M., Duarte M.M.M.F., de Freitas Bauermann L. (2018). The in vitro radiosensitizer potential of resveratrol on MCF-7 breast cancer cells. Chem. Biol. Interact..

[25] Tomé-Carneiro J., Gonzálvez M., Larrosa M., Yáñez-Gascón M.J., García-Almagro F.J., Ruiz-Ros J.A., Tomás-Barberán F.A., García-Conesa M.T., Espín J.C. (2013). Grape resveratrol increases serum adiponectin and downregulates inflammatory genes in peripheral blood mononuclear cells: A triple-blind, placebo-controlled, one-year clinical trial in patients with stable coronary artery disease. Cardiovasc. Drugs. Ther..

[26] Anthwal A., Thakur B.K., Rawat M., Rawat D., Tyagi A.K., Aggarwal B.B. (2014). Synthesis, characterization and in vitro anticancer activity of C-5 curcumin analogues with potential to inhibit TNF-α-induced NF-κB activation. BioMed Res. Int..

[27] Karthika C., Hari B., Mano V., Radhakrishnan A., Janani S., Akter R., Kaushik D., Rahman M.H. (2021). Curcumin as a great contributor for the treatment and mitigation of colorectal cancer. Exp. Gerontol..

[28] Abdulghani J., Gu L., Dagvadorj A., Lutz J., Leiby B., Bonuccelli G., Lisanti M.P., Zellweger T., Alanen K., Mirtti T.J.T.A. (2008). Stat3 promotes metastatic progression of prostate cancer. Am. J. Pathol..

[29] Lee J.-Y., Lee Y.-M., Chang G.-C., Yu S.-L., Hsieh W.-Y., Chen J.J., Chen H.-W., Yang P.-C.J.P. (2011). Curcumin induces EGFR degradation in lung adenocarcinoma and modulates p38 activation in intestine: The versatile adjuvant for gefitinib therapy. PLoS ONE.

[30] Kabir M., Rahman M., Akter R., Behl T., Kaushik D., Mittal V., Pandey P., Akhtar M.F., Saleem A., Albadrani G.M. (2021). Potential Role of Curcumin and Its Nanoformulations to Treat Various Types of Cancers. Biomolecules.

[31] Davie J.R., He S., Li L., Sekhavat A., Espino P., Drobic B., Dunn K.L., Sun J.-M., Chen H.Y., Yu J.J.A. (2008). Nuclear organization and chromatin dynamics–Sp1, Sp3 and histone deacetylases. Adv. Enzym. Regul..

[32] Akter R., Rahman H., Behl T., Chowdhury M., Rahman A., Manirujjaman M., Bulbul I.J., Elshenaw S.E., Tit D.M., Bungau S. (2020). Prospective role of polyphenolic compounds in the treatment of neurodegenerative diseases. CNS Neurol. Disord. Drug Targets..

[33] Wilken R., Veena M.S., Wang M.B., Srivatsan E.S. (2011). Curcumin: A review of anti-cancer properties and therapeutic activity in head and neck squamous cell carcinoma. Mol. Cancer.

[34] Bhattacharya T., Dutta S., Akter R., Rahman M., Karthika C., Nagaswarupa H.P., Murthy H.C.A., Fratila O., Brata R., Bungau S. (2021). Role of Phytonutrients in Nutrigenetics and Nutrigenomic Perspective in Curing Breast Cancer. Biomolecules.

[35] Gupta S.C., Patchva S., Koh W., Aggarwal B.B. (2012). Discovery of curcumin, a component of golden spice, and its miraculous biological activities. Clin. Exp. Pharmacol. Physiol..

[36] Ravindran J., Prasad S., Aggarwal B.B. (2009). Curcumin and cancer cells: How many ways can curry kill tumor cells selectively?. AAPS J..

[37] Sharma R.A., Euden S.A., Platton S.L., Cooke D.N., Shafayat A., Hewitt H.R., Marczylo T.H., Morgan B., Hemingway D., Plummer S.M. (2004). Phase I clinical trial of oral curcumin: Biomarkers of systemic activity and compliance. Clin. Cancer Res..

[38] Dhillon N., Aggarwal B.B., Newman R.A., Wolff R.A., Kunnumakkara A.B., Abbruzzese J.L., Ng C.S., Badmaev V., Kurzrock R. (2008). Phase II trial of curcumin in patients with advanced pancreatic cancer. Clin. Cancer Res..

[39] Hsieh C. (2001). Phase I clinical trial of curcumin, a chemopreventive agent, in patients with high-risk or pre-malignant lesions. Anticancer Res..

[40] Sharma R.A., McLelland H.R., Hill K.A., Ireson C.R., Euden S.A., Manson M.M., Pirmohamed M., Marnett L.J., Gescher A.J., Steward W.P. (2001). Pharmacodynamic and pharmacokinetic study of oral Curcuma extract in patients with colorectal cancer. Clin. Cancer Res..

[41] Asai A., Miyazawa T. (2000). Occurrence of orally administered curcuminoid as glucuronide and glucuronide/sulfate conjugates in rat plasma. Life Sci..

[42] (1991). European Union (EU) Council Directive 91/676/EEC of 12 December 1991 Concerning the Protection of Waters against Pollution Caused by Nitrates from Agricultural Sources. Eur. Union Bruss. Belg..

[43] Cruz–Correa M., Shoskes D.A., Sanchez P., Zhao R., Hylind L.M., Wexner S.D., Giardiello F.M. (2006). Combination treatment with curcumin and quercetin of adenomas in familial adenomatous polyposis. Clin. Gastroenterol. Hepatol..

[44] Carroll R.E., Benya R.V., Turgeon D.K., Vareed S., Neuman M., Rodriguez L., Kakarala M., Carpenter P.M., McLaren C., Meyskens F.L. (2011). Phase IIa clinical trial of curcumin for the prevention of colorectal neoplasia. Cancer Prev. Res..

[45] Kanai M., Yoshimura K., Asada M., Imaizumi A., Suzuki C., Matsumoto S., Nishimura T., Mori Y., Masui T., Kawaguchi Y. (2011). A phase I/II study of gemcitabine-based chemotherapy plus curcumin for patients with gemcitabine-resistant pancreatic cancer. Cancer Chemother. Pharmacol..

[46] Bayet-Robert M., Kwiatowski F., Leheurteur M., Gachon F., Planchat E., Abrial C., Mouret-Reynier M.-A., Durando X., Barthomeuf C., Chollet P. (2010). Phase I dose escalation trial of docetaxel plus curcumin in patients with advanced and metastatic breast cancer. Cancer Biol. Ther..

[47] Antunes L.M.G., Araújo M.C.P., Darin J.D.A.C., Maria de Lourdes P.B.J.M.R.G.T., Mutagenesis E. (2000). Effects of the antioxidants curcumin and vitamin C on cisplatin-induced clastogenesis in Wistar rat bone marrow cells. Mutat. Res. Genet. Toxicol. Environ. Mutagen..

[48] Liu Y.-Q., Wang X.-L., He D.-H., Cheng Y.-X. (2020). Protection against chemotherapy-and radiotherapy-induced side effects: A review based on the mechanisms and therapeutic opportunities of phytochemicals. Phytomedicine.

[49] Holick M.F. (2006). Vitamin D: Its role in cancer prevention and treatment. Prog. Biophys. Mol. Biol..

[50] Lazarus H., Haynesworth S., Gerson S., Rosenthal N., Caplan A. (1995). Ex vivo expansion and subsequent infusion of human bone marrow-derived stromal progenitor cells (mesenchymal progenitor cells): Implications for therapeutic use. Bone Marrow Transplant..

[51] Rosen C.J. (2011). Vitamin D insufficiency. N. Engl. J. Med..

[52] Plum L.A., DeLuca H.F. (2009). The functional metabolism and molecular biology of vitamin D action. Clin. Cases. Miner. Bone Metab..

[53] Norman A.W., Bouillon R. (2010). Vitamin D nutritional policy needs a vision for the future. Exp. Biol. Med..

[54] Feldman D., Krishnan A.V., Swami S., Giovannucci E., Feldman B.J. (2014). The role of vitamin D in reducing cancer risk and progression. Nat. Rev. Cancer.

[55] Ingraham B.A., Bragdon B., Nohe A. (2008). Molecular basis of the potential of vitamin D to prevent cancer. Curr. Med. Res. Opin..

[56] Masuda S., Jones G. (2006). Promise of vitamin D analogues in the treatment of hyperproliferative conditions. Mol. Cancer Ther..

[57] Bouillon R., Carmeliet G., Verlinden L., van Etten E., Verstuyf A., Luderer H.F., Lieben L., Mathieu C., Demay M. (2008). Vitamin D and human health: Lessons from vitamin D receptor null mice. Endocr. Rev..

[58] Cihan Y.B. (2019). Does vitamin D prevent radiotherapy-induced toxicity?. Turkish J. Biochem..

[59] Parrón T., Requena M., Hernández A.F., Alarcón R. (2014). Environmental exposure to pesticides and cancer risk in multiple human organ systems. Toxicol. Lett..

[60] Cui Y., Rohan T.E. (2006). Vitamin D, calcium, and breast cancer risk: A review. Cancer Epidemiol. Biomark. Prev..

[61] John E.M., Koo J., Schwartz G.G. (2007). Sun exposure and prostate cancer risk: Evidence for a protective effect of early-life exposure. Cancer Epidemiol. Biomark. Prev..

[62] Gupta D., Lammersfeld C., Trukova K., Lis C. (2009). Vitamin D and prostate cancer risk: A review of the epidemiological literature. Prostate Cancer Prostatic Dis..

[63] Waltz P., Chodick G. (2008). Assessment of ecological regression in the study of colon, breast, ovary, non-Hodgkin’s lymphoma, or prostate cancer and residential UV. Eur. J. Cancer Prev..

[64] Wang J., Jiang Y.-F. (2012). Natural compounds as anticancer agents: Experimental evidence. World J. Exp. Med..

[65] Hathcock J.N., Shao A., Vieth R., Heaney R. (2007). Risk assessment for vitamin D. Am. J. Clin. Nutr..

[66] Jones G. (2008). Pharmacokinetics of vitamin D toxicity. Am. J. Clin. Nutr..

[67] Ma Y., Khalifa B., Yee Y.K., Lu J., Memezawa A., Savkur R.S., Yamamoto Y., Chintalacharuvu S.R., Yamaoka K., Stayrook K.R. (2006). Identification and characterization of noncalcemic, tissue-selective, nonsecosteroidal vitamin D receptor modulators. J. Clin. Investig..

[68] Beer T.M., Lemmon D., Lowe B.A., Henner W.D. (2003). High-dose weekly oral calcitriol in patients with a rising PSA after prostatectomy or radiation for prostate carcinoma. Cancer Interdiscip. Int. J. Am. Cancer Soc..

[69] Trump D.L., Potter D.M., Muindi J., Brufsky A., Johnson C.S. (2006). Phase II trial of high-dose, intermittent calcitriol (1, 25 dihydroxyvitamin D3) and dexamethasone in androgen-independent prostate cancer. Cancer.

[70] Zhou P., Yang X.-L., Wang X.-G., Hu B., Zhang L., Zhang W., Si H.-R., Zhu Y., Li B., Huang C.-L. (2020). A pneumonia outbreak associated with a new coronavirus of probable bat origin. Nature.

[71] Bufu T., Di X., Yilin Z., Gege L., Xi C., Ling W.J. (2018). Celastrol inhibits colorectal cancer cell proliferation and migration through suppression of MMP3 and MMP7 by the PI3K/AKT signaling pathway. Anticancer Drugs.

[72] Wang G., Fersht A.R. (2017). Multisite aggregation of p53 and implications for drug rescue. Proc. Natl. Acad. Sci. USA.

[73] Huang Y., Zhou Y., Fan Y., Zhou D.J. (2008). Celastrol inhibits the growth of human glioma xenografts in nude mice through suppressing VEGFR expression. Cancer Lett..

[74] Lee J.-H., Choi K.J., Seo W.D., Jang S.Y., Kim M., Lee B.W., Kim J.Y., Kang S., Park K.H., Lee Y.-S. (2011). Enhancement of radiation sensitivity in lung cancer cells by celastrol is mediated by inhibition of Hsp90. Int. J. Mol. Med..

[75] Seo H.R., Seo W.D., Pyun B.-J., Lee B.W., Jin Y.B., Park K.H., Seo E.-K., Lee Y.-J., Lee Y.-S. (2011). Radiosensitization by celastrol is mediated by modification of antioxidant thiol molecules. Chem. Biol. Interact..

[76] Jun H.Y., Kim T.-H., Choi J.W., Lee Y.H., Lee K.K., Yoon K.-H. (2017). Evaluation of connectivity map-discovered celastrol as a radiosensitizing agent in a murine lung carcinoma model: Feasibility study of diffusion-weighted magnetic resonance imaging. PLoS ONE.

[77] Fusi F., Durante M., Sgaragli G., Khanh P.N., Huong T.T., Cuong N.M. (2015). In vitro vasoactivity of zerumbone from Zingiber zerumbet. Planta Med..

[78] Yob N., Jofrry S.M., Affandi M., Teh L., Salleh M., Zakaria Z. (2011). Zingiber zerumbet (L.): A review of its ethnomedicinal, chemical, and pharmacological uses. Evid. Based Complementary Altern. Med..

[79] Rahman H.S., Rasedee A., Yeap S.K., Othman H.H., Chartrand M.S., Namvar F., Abdul A.B., How C.W. (2014). Biomedical properties of a natural dietary plant metabolite, zerumbone, in cancer therapy and chemoprevention trials. BioMed Res. Int..

[80] Murakami A., Tanaka T., Lee J.Y., Surh Y.J., Kim H.W., Kawabata K., Nakamura Y., Jiwajinda S., Ohigashi H. (2004). Zerumbone, a sesquiterpene in subtropical ginger, suppresses skin tumor initiation and promotion stages in ICR mice. Int. J. Cancer.

[81] Sung B., Jhurani S., Ahn K.S., Mastuo Y., Yi T., Guha S., Liu M., Aggarwal B.B. (2008). Zerumbone down-regulates chemokine receptor CXCR4 expression leading to inhibition of CXCL12-induced invasion of breast and pancreatic tumor cells. Cancer Res..

[82] Choi S.-H., Lee Y.-J., Seo W.D., Lee H.-J., Nam J.-W., Lee Y.J., Kim J., Seo E.-K., Lee Y.-S. (2011). Altered cross-linking of HSP27 by zerumbone as a novel strategy for overcoming HSP27-mediated radioresistance. Int. J. Radiat. Oncol. Biol. Phys..

[83] Huang G.-C., Chien T.-Y., Chen L.-G., Wang C.-C. (2005). Antitumor effects of zerumbone from Zingiber zerumbet in P-388D1 cells in vitro and in vivo. Planta Med..

[84] Chiang P.-K., Tsai W.-K., Chen M., Lin W.-R., Chow Y.-C., Lee C.-C., Hsu J.-M., Chen Y.-J. (2018). Zerumbone regulates DNA repair responding to Ionizing radiation and enhances radiosensitivity of human prostatic cancer cells. Integr. Cancer Ther..

[85] Bousselham A., Bouattane O., Youssfi M., Raihani A.J. (2018). Brain tumor temperature effect extraction from MRI imaging using bioheat equation. Procedia Comput. Sci..

[86] Kansal A.R., Torquato S., Harsh G., Chiocca E., Deisboeck T.J. (2000). Simulated brain tumor growth dynamics using a three-dimensional cellular automaton. J. Theor. Biol..

[87] Weng H.-Y., Hsu M.-J., Wang C.-C., Chen B.-C., Hong C.-Y., Chen M.-C., Chiu W.-T., Lin C.-H. (2012). Zerumbone suppresses IKKα, Akt, and FOXO1 activation, resulting in apoptosis of GBM 8401 cells. J. Biomed. Sci..

[88] Woźniak Ł., Skąpska S., Marszałek K. (2015). Ursolic acid—A pentacyclic triterpenoid with a wide spectrum of pharmacological activities. Molecules.

[89] Koh S.J., Tak J.K., Kim S.T., Nam W.S., Kim S.Y., Park K.M., Park J.-W. (2012). Sensitization of ionizing radiation-induced apoptosis by ursolic acid. Free Radic. Res..

[90] Lee Y.-H., Wang E., Kumar N., Glickman R.D. (2014). Ursolic acid differentially modulates apoptosis in skin melanoma and retinal pigment epithelial cells exposed to UV–VIS broadband radiation. Apoptosis.

[91] Song B., Zhang Q., Yu M., Qi X., Wang G., Xiao L., Yi Q., Jin W. (2017). Ursolic acid sensitizes radioresistant NSCLC cells expressing HIF-1α through reducing endogenous GSH and inhibiting HIF-1α. Oncol. Lett..

[92] Wu D.M., Lu J., Zhang Y.Q., Zheng Y.L., Hu B., Cheng W., Zhang Z.-F., Li M.Q. (2013). Ursolic acid improves domoic acid-induced cognitive deficits in mice. Toxicol. Appl. Pharmacol..

[93] Lu J., Wu D.-M., Zheng Y.-L., Hu B., Zhang Z.-F., Ye Q., Liu C.-M., Shan Q., Wang Y.-J. (2010). Ursolic acid attenuates D-galactose-induced inflammatory response in mouse prefrontal cortex through inhibiting AGEs/RAGE/NF-κB pathway activation. Cereb. Cortex..

[94] Kupchan S.M., Doskotch R.W., Bollinger P., McPhail A., Sim G., Renauld J.S. (1965). The Isolation and Structural Elucidation of a Novel Steroidal Tumor Inhibitor from Acnistus arborescens1, 2. J. Am. Chem. Soc..

[95] Shohat B., Gitter S., Abraham A., Lavie D. (1967). Antitumor activity of withaferin A (NSC-101088). Cancer Chemother. Rep..

[96] Lee I.-C., Choi B.Y. (2016). Withaferin-A—A natural anticancer agent with pleitropic mechanisms of action. Int. J. Mol. Sci..

[97] Sharada A.C., Solomon F.E., Devi P.U., Udupa N., Srinivasan K.K. (1996). Antitumor and radiosensitizing effects of withaferin A on mouse Ehrlich ascites carcinoma in vivo. Acta Oncol..

[98] Kamath R., Rao B.S., Devi P.U. (1999). Response of a mouse fibrosarcoma to withaferin A and radiation. Pharm. Pharmacol. Commun..

[99] Murata R., Siemann D.W., Overgaard J., Horsman M.R. (2001). Improved tumor response by combining radiation and the vascular-damaging drug 5, 6-dimethylxanthenone-4-acetic acid. Radiat. Res..

[100] Oh J.H., Lee T.-J., Kim S.H., Choi Y.H., Lee S.H., Lee J.M., Kim Y.-H., Park J.-W., Kwon T.K. (2008). Induction of apoptosis by withaferin A in human leukemia U937 cells through down-regulation of Akt phosphorylation. Apoptosis.

[101] Yang E.S., Choi M.J., Kim J.H., Choi K.S., Kwon T.K. (2011). Combination of withaferin A and X-ray irradiation enhances apoptosis in U937 cells. Toxicol. Vitr..

[102] Yang E.S., Choi M.J., Kim J.H., Choi K.S., Kwon T.K. (2011). Withaferin A enhances radiation-induced apoptosis in Caki cells through induction of reactive oxygen species, Bcl-2 downregulation and Akt inhibition. Chem. Biol. Interact..

[103] Widodo N., Kaur K., Shrestha B.G., Takagi Y., Ishii T., Wadhwa R., Kaul S.C. (2007). Selective killing of cancer cells by leaf extract of Ashwagandha: Identification of a tumor-inhibitory factor and the first molecular insights to its effect. Clin. Cancer Res..

[104] Hahm E.-R., Moura M.B., Kelley E.E., Van Houten B., Shiva S., Singh S.V. (2011). Withaferin A-induced apoptosis in human breast cancer cells is mediated by reactive oxygen species. PLoS ONE.

[105] Sehrawat A., Samanta S.K., Hahm E.-R., Croix C.S., Watkins S., Singh S.V. (2019). Withaferin A-mediated apoptosis in breast cancer cells is associated with alterations in mitochondrial dynamics. Mitochondrion.

[106] Li L., Tian Y., Yu J., Song X., Jia R., Cui Q., Tong W., Zou Y., Li L., Yin L. (2017). iTRAQ-based quantitative proteomic analysis reveals multiple effects of Emodin to Haemophilus parasuis. J. Proteomics.

[107] Chen T., Zheng L.Y., Xiao W., Gui D., Wang X., Wang N. (2015). Emodin ameliorates high glucose induced-podocyte epithelial-mesenchymal transition in-vitro and in-vivo. Cell. Physiol. Biochem..

[108] Liu Y., Hou H., Li D., Cheng D., Qin C., Li W. (2010). Enhancement effect of emodin on radiosensitivity of human nasopharyngeal carcinoma transplanted in nude mice. Chin. Pharm. J..

[109] Shrimali D., Shanmugam M.K., Kumar A.P., Zhang J., Tan B.K., Ahn K.S., Sethi G. (2013). Targeted abrogation of diverse signal transduction cascades by emodin for the treatment of inflammatory disorders and cancer. Cancer Lett..

[110] Dey D., Ray R., Hazra B. (2014). Antitubercular and antibacterial activity of quinonoid natural products against multi-drug resistant clinical isolates. Phytother. Res..

[111] Gu J., Cui C.-F., Yang L., Wang L., Jiang X.-H. (2019). Emodin Inhibits Colon Cancer Cell Invasion and Migration by Suppressing Epithelial-Mesenchymal Transition via the Wnt/β-Catenin Pathway. Oncol. Res. Featur. Preclin. Clin. Cancer Ther..

[112] Luo J., Yuan Y., Chang P., Li D., Liu Z., Qu Y. (2014). Combination of aloe-emodin with radiation enhances radiation effects and improves differentiation in human cervical cancer cells. Mol. Med. Rep..

[113] Miller R.C., Murley J.S., Rademaker A.W., Woloschak G.E., Li J.J., Weichselbaum R.R., Grdina D.J. (2016). Very low doses of ionizing radiation and redox associated modifiers affect survivin-associated changes in radiation sensitivity. Free Radic. Biol. Med..

[114] Chen R.-S., Jhan J.-Y., Su Y.-J., Lee W.-T., Cheng C.-M., Ciou S.-C., Lin S.-T., Chuang S.-M., Ko J.-C., Lin Y.-W. (2009). Emodin enhances gefitinib-induced cytotoxicity via Rad51 downregulation and ERK1/2 inactivation. Exp. Cell Res..

[115] Lai J.-M., Chang J.T., Wen C.-L., Hsu S.-L. (2009). Emodin induces a reactive oxygen species-dependent and ATM-p53-Bax mediated cytotoxicity in lung cancer cells. Eur. J. Pharmacol..

[116] Ko J.-C., Su Y.-J., Lin S.-T., Jhan J.-Y., Ciou S.-C., Cheng C.-M., Chiu Y.-F., Kuo Y.-H., Tsai M.-S., Lin Y.-W. (2010). Emodin enhances cisplatin-induced cytotoxicity via down-regulation of ERCC1 and inactivation of ERK1/2. Lung Cancer.

[117] Kong W., Wei J., Abidi P., Lin M., Inaba S., Li C., Wang Y., Wang Z., Si S., Pan H. (2004). Berberine is a novel cholesterol-lowering drug working through a unique mechanism distinct from statins. Nat. Med..

[118] Yin J., Xing H., Ye J. (2008). Efficacy of berberine in patients with type 2 diabetes mellitus. Metabolism.

[119] Liu Z., Liu Q., Xu B., Wu J., Guo C., Zhu F., Yang Q., Gao G., Gong Y., Shao C. (2009). Berberine induces p53-dependent cell cycle arrest and apoptosis of human osteosarcoma cells by inflicting DNA damage. Mutat. Res. Fundam. Mol. Mech. Mutagenesis.

[120] Lin J.-P., Yang J.-S., Lee J.-H., Hsieh W.-T., Chung J.-G. (2006). Berberine induces cell cycle arrest and apoptosis in human gastric carcinoma SNU-5 cell line. World J. Gastroenterol..

[121] Hwang J.-M., Kuo H.-C., Tseng T.-H., Liu J.-Y., Chu C.-Y. (2006). Berberine induces apoptosis through a mitochondria/caspases pathway in human hepatoma cells. Arch. Toxicol..

[122] Peng P.-l., Kuo W.-H., Tseng H.-C., Chou F.-P. (2008). Synergistic tumor-killing effect of radiation and berberine combined treatment in lung cancer: The contribution of autophagic cell death. Int. J. Radiat. Oncol. Biol. Phys..

[123] Liu Q., Jiang H., Liu Z., Wang Y., Zhao M., Hao C., Feng S., Guo H., Xu B., Yang Q. (2011). Berberine radiosensitizes human esophageal cancer cells by downregulating homologous recombination repair protein RAD51. PLoS ONE.

[124] Rosser C.J., Tanaka M., Pisters L.L., Tanaka N., Levy L.B., Hoover D.C., Grossman H.B., McDonnell T.J., Kuban D.A., Meyn R.E. (2004). Adenoviral-mediated PTEN transgene expression sensitizes Bcl-2-expressing prostate cancer cells to radiation. Cancer Gene Ther..

[125] Szotowski B., Antoniak S., Goldin-Lang P., Tran Q.-V., Pels K., Rosenthal P., Bogdanov V.Y., Borchert H.-H., Schultheiss H.-P., Rauch U. (2007). Antioxidative treatment inhibits the release of thrombogenic tissue factor from irradiation-and cytokine-induced endothelial cells. Cardiovasc. Res..

[126] Böhnke A., Westphal F., Schmidt A., El-Awady R., Dahm-Daphi J. (2004). Role of p53 mutations, protein function and DNA damage for the radiosensitivity of human tumour cells. Int. J. Radiat. Biol..

[127] Zhang Y., Chen F. (2004). Reactive oxygen species (ROS), troublemakers between nuclear factor-κB (NF-κB) and c-Jun NH2-terminal kinase (JNK). Cancer Res..

[128] Wang J., Liu Q., Yang Q. (2012). Radiosensitization effects of berberine on human breast cancer cells. Int. J. Mol. Med..

[129] Kawano M., Takagi R., Kaneko A., Matsushita S.J. (2015). Berberine is a dopamine D1-and D2-like receptor antagonist and ameliorates experimentally induced colitis by suppressing innate and adaptive immune responses. J. Neuroimmunol..

[130] Li H., Li X.L., Zhang M., Xu H., Wang C.C., Wang S., Duan R.S. (2014). Berberine ameliorates experimental autoimmune neuritis by suppressing both cellular and humoral immunity. Scand. J. Immunol..

[131] Wang Y.X., Pang W.Q., Zeng Q.X., Deng Z.S., Fan T.Y., Jiang J.D., Deng H.B., Song D.Q. (2018). Synthesis and biological evaluation of new berberine derivatives as cancer immunotherapy agents through targeting IDO1. Eur. J. Med. Chem..

[132] Kieliszek M., Lipinski B. (2018). Pathophysiological significance of protein hydrophobic interactions: An emerging hypothesis. Med. Hypotheses.

[133] Kieliszek M., Lipinski B., Błażejak S. (2017). Application of sodium selenite in the prevention and treatment of cancers. Cells.

[134] Liu T., Shi C., Duan L., Zhang Z., Luo L., Goel S., Cai W., Chen T. (2018). A highly hemocompatible erythrocyte membrane-coated ultrasmall selenium nanosystem for simultaneous cancer radiosensitization and precise antiangiogenesis. J. Mater. Chem. B.

[135] Wang M., Law M.E., Castellano R.K., Law B.K. (2018). The unfolded protein response as a target for anticancer therapeutics. Crit. Rev. Oncol..

[136] Spagnuolo C., Russo G.L., Orhan I.E., Habtemariam S., Daglia M., Sureda A., Nabavi S.F., Devi K.P., Loizzo M.R., Tundis R. (2015). Genistein and cancer: Current status, challenges, and future directions. Adv. Nutr..

[137] Uifălean A., Schneider S., Ionescu C., Lalk M., Iuga C.A. (2016). Soy isoflavones and breast cancer cell lines: Molecular mechanisms and future perspectives. Molecules.

[138] Banerjee S., Li Y., Wang Z., Sarkar F.H. (2008). Multi-targeted therapy of cancer by genistein. Cancer Lett..

[139] Shi Y. (2002). Mechanisms of caspase activation and inhibition during apoptosis. Mol. Cell.

[140] Altieri D.C. (2003). Validating survivin as a cancer therapeutic target. Nat. Rev. Cancer.

[141] Zhang B., Liu J.-y., Pan J.-s., Han S.-p., Yin X.-x., Wang B., Hu G. (2006). Combined treatment of ionizing radiation with genistein on cervical cancer HeLa cells. J. Pharmacol. Sci..

[142] Yashar C.M., Spanos W.J., Taylor D.D., Gercel-Taylor C. (2005). Potentiation of the radiation effect with genistein in cervical cancer cells. Gynecol. Oncol..

[143] Wang S., Yang K., Hsu Y., Chang C., Yang Y. (2001). The differential inhibitory effects of genistein on the growth of cervical cancer cells in vitro. Neoplasma.

[144] Liu H.-Y., Skjetne E., Kobernus M. (2013). Mobile phone tracking: In support of modelling traffic-related air pollution contribution to individual exposure and its implications for public health impact assessment. Environ. Health.

[145] Xie Q., Bai Q., Zou L.Y., Zhang Q.Y., Zhou Y., Chang H., Yi L., Zhu J.D., Mi M.T. (2014). Genistein inhibits DNA methylation and increases expression of tumor suppressor genes in human breast cancer cells. Genes Chromosomes Cancer.

[146] Majid S., Dar A.A., Shahryari V., Hirata H., Ahmad A., Saini S., Tanaka Y., Dahiya A.V., Dahiya R. (2010). Genistein reverses hypermethylation and induces active histone modifications in tumor suppressor gene B-Cell translocation gene 3 in prostate cancer. Cancer Interdiscip. Int. J. Am. Cancer Soc..

[147] Baird L., Llères D., Swift S., Dinkova-Kostova A.T. (2013). Regulatory flexibility in the Nrf2-mediated stress response is conferred by conformational cycling of the Keap1-Nrf2 protein complex. Proc. Natl. Acad. Sci. USA.

[148] Cho H.-Y., Reddy S.P., DeBiase A., Yamamoto M., Kleeberger S.R. (2005). Gene expression profiling of NRF2-mediated protection against oxidative injury. Free Radic. Biol. Med..

[149] Liu X., Sun C., Liu B., Jin X., Li P., Zheng X., Zhao T., Li F., Li Q. (2016). Genistein mediates the selective radiosensitizing effect in NSCLC A549 cells via inhibiting methylation of the keap1 gene promoter region. Oncotarget.

[150] You S., Li R., Park D., Xie M., Sica G.L., Cao Y., Xiao Z.-Q., Deng X. (2014). Disruption of STAT3 by niclosamide reverses radioresistance of human lung cancer. Mol. Cancer Ther..

[151] Du Y., Ji X. (2014). Bcl-2 down-regulation by small interfering RNA induces Beclin1-dependent autophagy in human SGC-7901 cells. Cell Biol. Int..

[152] Pattingre S., Tassa A., Qu X., Garuti R., Liang X.H., Mizushima N., Packer M., Schneider M.D., Levine B. (2005). Bcl-2 antiapoptotic proteins inhibit Beclin 1-dependent autophagy. Cell.

[153] Zhang Z., Jin F., Lian X., Li M., Wang G., Lan B., He H., Liu G.-D., Wu Y., Sun G. (2018). Genistein promotes ionizing radiation-induced cell death by reducing cytoplasmic Bcl-xL levels in non-small cell lung cancer. Sci. Rep..

[154] Sahin K., Yenice E., Bilir B., Orhan C., Tuzcu M., Sahin N., Ozercan I.H., Kabil N., Ozpolat B., Kucuk O.J. (2019). Genistein prevents development of spontaneous ovarian cancer and inhibits tumor growth in hen model. Cancer Prev. Res..

[155] Hsiao Y.C., Peng S.F., Lai K.C., Liao C.L., Huang Y.P., Lin C.C., Lin M.L., Liu K.C., Tsai C.C., Ma Y.S. (2019). Genistein induces apoptosis in vitro and has antitumor activity against human leukemia HL-60 cancer cell xenograft growth in vivo. Environ. Toxicol..

[156] Holsti L.R. (1995). Development of clinical radiotherapy since 1896. Acta Oncol..

[157] Gai S., Yang G., Yang P., He F., Lin J., Jin D., Xing B. (2018). Recent advances in functional nanomaterials for light–triggered cancer therapy. Nano Today.

[158] Alberti C. (2011). Organ-confined prostate carcinoma radiation brachytherapy compared with external either photon-or hadron-beam radiation therapy. Just a short up-to-date. Eur. Rev. Med. Pharmacol. Sci..

[159] Islam M.A., Islam S., Akter A., Rahman M.H., Nandwani D. (2017). Effect of organic and inorganic fertilizers on soil properties and the growth, yield and quality of tomato in Mymensingh, Bangladesh. Agriculture.

[160] Malfa G.A., Tomasello B., Acquaviva R., Genovese C., La Mantia A., Cammarata F.P., Ragusa M., Renis M., Di Giacomo C. (2019). Betula etnensis Raf. (Betulaceae) extract induced HO-1 expression and ferroptosis cell death in human colon cancer cells. Int. J. Mol. Sci..

[161] Reed D., Raina K., Agarwal R. (2018). Nutraceuticals in prostate cancer therapeutic strategies and their neo-adjuvant use in diverse populations. NPJ Precis. Oncol..

[162] Das L., Bhaumik E., Raychaudhuri U., Chakraborty R. (2012). Role of nutraceuticals in human health. J. Food Sci. Technol..

[163] Johnson G.E., Ivanov V.N., Hei T.K. (2008). Radiosensitization of melanoma cells through combined inhibition of protein regulators of cell survival. Apoptosis.

[164] Minafra L., Porcino N., Bravatà V., Gaglio D., Bonanomi M., Amore E., Cammarata F.P., Russo G., Militello C., Savoca G. (2019). Radiosensitizing effect of curcumin-loaded lipid nanoparticles in breast cancer cells. Sci. Rep..

[165] Sandur S.K., Deorukhkar A., Pandey M.K., Pabón A.M., Shentu S., Guha S., Aggarwal B.B., Krishnan S. (2009). Curcumin modulates the radiosensitivity of colorectal cancer cells by suppressing constitutive and inducible NF-κB activity. Int. J. Radiat. Oncol. Biol. Phys..

[166] Spina C., Tangpricha V., Yao M., Zhou W., Wolfe M., Maehr H., Uskokovic M., Adorini L., Holick M.J. (2005). Colon cancer and solar ultraviolet B radiation and prevention and treatment of colon cancer in mice with vitamin D and its Gemini analogs. J. Steroid. Biochem. Mol. Biol..

[167] Chlebowski R.T., Johnson K.C., Kooperberg C., Pettinger M., Wactawski-Wende J., Rohan T., Rossouw J., Lane D., O’Sullivan M.J., Yasmeen S.J. (2008). Calcium plus vitamin D supplementation and the risk of breast cancer. J. Natl. Cancer Inst..

[168] Dai Y., DeSano J.T., Meng Y., Ji Q., Ljungman M., Lawrence T.S., Xu L. (2009). Celastrol potentiates radiotherapy by impairment of DNA damage processing in human prostate cancer. Int. J. Radiat. Oncol. Biol. Phys..

[169] Chiang M.-F., Chen H.-H., Chi C.-W., Sze C.-I., Hsu M.-L., Shieh H.-R., Lin C.-P., Tsai J.-T., Chen Y.-J. (2015). Modulation of Sonic hedgehog signaling and WW domain containing oxidoreductase WOX1 expression enhances radiosensitivity of human glioblastoma cells. Exp. Biol. Med..

[170] Deorukhkar A., Ahuja N., Mercado A.L., Diagaradjane P., Raju U., Patel N., Mohindra P., Diep N., Guha S., Krishnan S. (2015). Zerumbone increases oxidative stress in a thiol-dependent ROS-independent manner to increase DNA damage and sensitize colorectal cancer cells to radiation. Cancer Med..

[171] Yang Y., Jiang M., Hu J., Lv X., Yu L., Qian X., Liu B. (2015). Enhancement of radiation effects by ursolic acid in BGC-823 human adenocarcinoma gastric cancer cell line. PLoS ONE.

[172] Hur J., Kim D. (2010). Berberine inhibited radioresistant effects and enhanced anti-tumor effects in the irradiated-human prostate cancer cells. Toxicol. Res..

